# Factors Associated with HIV Status Disclosure and Its Effect on Treatment Adherence and Quality of Life among Children 6–17 Years on Antiretroviral Therapy in Southern Highlands Zone, Tanzania: Unmatched Case Control Study

**DOI:** 10.1155/2018/8058291

**Published:** 2018-06-26

**Authors:** Regina Edward Bulali, Stephen Matthew Kibusi, Bonaventura C. T. Mpondo

**Affiliations:** ^1^School of Nursing and Public Health, College of Health Science, University of Dodoma, Dodoma, Tanzania; ^2^School of Medicine and Dentistry, College of Health Science, University of Dodoma, Dodoma, Tanzania

## Abstract

**Background:**

The World Health Organization (WHO) recommends that children should be informed of their HIV status at ages 6 to 12 years and full disclosure of HIV and AIDS be offered in a caring and supportive manner at about 8 to 10 years. The objective of this study was to determine factors associated with HIV status disclosure and its effect on treatment adherence and health-related quality of life among children between 6 and 17 years of age living with HIV/AIDS in the Southern Highlands Zone, Tanzania, 2017.

**Methods:**

A hospital based unmatched case control study was conducted between April and September 2017. A total of 309 children between 6 and 17 years on ART for at least six months were enrolled in this study. Simple random sampling was employed in selecting the children from existing treatment registers. Data were collected using a structured questionnaire which included the WHO Quality of Life standard tool (WHOQOL-BREF 2012 tool) and treatment adherence manual. Multiple logistic regression was used to test for the independent effect of HIV status disclosure on treatment adherence and quality of life at p value less than 0.05.

**Results:**

Out of 309 children, only 102 (33%) had their HIV status disclosed to them. The mean age at HIV status disclosure was 12.39 (SD=3.015). HIV status disclosure was high among girls (51%), children aged 10-13 years (48.3%), and those living with their biological parents (59.8%). After adjusting for confounders, being aged between 10-13 and 14-17 years was associated with HIV status disclosure (AOR 19.178, p<0.05 and AOR=65.755, p<0.001, respectively). HIV status disclosure was associated with ART adherence (AOR=8.173, p<0.05) and increased the odds of having good quality of life (AOR=3.283, p<0.001).

**Conclusions:**

HIV status disclosure significantly improved adherence to treatment and quality of life among children living with HIV/AIDS.

## 1. Introduction

Globally, it is estimated that 36.7 million people live with HIV/AIDS. Of these, 1.8 million are children less than 15 years of age. In 2015, it was estimated that there were 150,000 children less than 15 years who became newly infected with HIV. Most of these children live in Sub-Saharan Africa and are infected by their HIV-positive mothers during pregnancy, childbirth, or breastfeeding [1].

Although there has been significant improvement in ART coverage among children, it is still low compared to adults. At the end of 2016, it was estimated that only 43% of children aged <15 years living with HIV/AIDS were receiving ART [2]. As the ART coverage continues to increase among children, the challenge of HIV status disclosure and treatment adherence will further grow. Evidence shows that adherence level of >95% is required to attain sustained virological suppression and better treatment outcomes.

In 2011, WHO released a guideline on HIV status disclosure in children [3]. The guideline recommends that disclosure process should start when the child is 6 years old and be completed at the age of 12 years. However, there are several reports of very low levels of disclosure especially in resource limited settings [4, 5]. In one systematic review, the level of HIV status disclosure was found to range from 0% to 69% [6]. Several barriers have been identified as to why there is low level of status disclosure among children. In a study done in Malawi, despite reported importance of disclosing HIV status to infected children, the parents/guardians felt unease and were in dilemma whether to disclose or not [7]. There is also evidence that parents/guardians opt not to disclose because they are not sure of the child's reaction after disclosure [5, 6].

There is evidence that HIV status disclosure is associated with improved health among children and halted disease progression [8]. However, there are mixed views on the association between disclosure and treatment adherence. In a recent review for the association between disclosure and treatment adherence, five of the reviewed papers showed that disclosure improved adherence; however there were four papers that showed a negative association between disclosure and adherence [9]. Therefore, there are mixed results from existing studies for the association between HIV status disclosure in children and treatment adherence. Association between HIV status disclosure and overall quality of life in HIV-infected children has not been well studied especially in developing countries where the burden is high. In this study we aimed at determining the factors associated with HIV status disclosure and its effect on treatment adherence and quality of life among children aged between 6 and 17 years in the Southern Highlands Zone, Tanzania.

## 2. Materials and Methods

### 2.1. Setting

This study was conducted in pediatric HIV care and treatment centres in Iringa and Mbeya regions, Southern Highlands Zone of Tanzania. The two regions have the highest prevalence of HIV in the country. The Iringa region borders the dry belt of central Tanzania in the north and south by Lake Nyasa. It lies between latitudes 7° 05° 32 and 12 South and longitude 33° 47° 32 to 36 east of Meridian. Iringa region is contiguous with the Dodoma and Singida regions in the north, Mbeya to the west, Morogoro in the east, and Ruvuma in the south. Lake Nyasa separates Iringa Region and Malawi in the southwestern Tanzania. It has four districts with a population of 941,238 (NBS, 2013).

The Mbeya region lies between latitude 70 and 90 31' south of the Equator and between longitude 320 and 350 east of Greenwich. Mbeya shares borders with the Republic of Malawi and Zambia to the south, Songwe Region to the west, Singida and Tabora regions to the north, and Iringa and Njombe regions to the east. The region has five districts with a total population of 2,707,410 people (NBS, 2013).

### 2.2. Research Design

This was an unmatched case control study. The chances that the controls could be healthier than cases were controlled by random selection of participants.

### 2.3. Study Population

The study population was children living with HIV/AIDS who stayed in Iringa or Mbeya region in Southern Highlands Zone, Tanzania. Inclusion criteria were HIV-infected children between 6 and 17 years of age on ART for not less than six months, who were attending pediatric HIV care and treatment centres in the Southern Highlands Zone, Tanzania. The age range from 6 to 17 years was selected because WHO 2011 recommends age 6 as a starting point for disclosure and age 17 is considered as childhood age before a child reaches 18 years.

### 2.4. Sample Size and Sampling Process

A sample size was 309 subjects, computed by using WINPEPI program (Abramson 2004, 2011) computer software. The data computed include difference between means, significance level = 5%, power = 80%, ratio B: A = 2, SD in A: 32, SD in B: 28, and difference = 10.

### 2.5. Expected Precision

Approximately 95% CI for difference between means (D) = D - 7.001 to D + 7.00.

Two regions (Mbeya and Iringa) among seven regions in Southern Highlands Zone were purposively selected because they had higher HIV prevalence. A simple random sampling using a lottery technique was used to select one district from each selected region whereby Mbeya city council and Iringa municipal district were selected. Then five CTC per district were purposively selected based on the number of clients they serve to ensure that the needed sample size could be attained. The required sample of participants was equally divided among selected centres. HIV-infected children attending services from pediatric HIV care and treatment centres of selected hospitals from June 2016 six months before the survey were identified from the registers. Then, using the patients register, cards, and files, children on ART for at least six months were randomly enrolled to the study. Thereafter, caregivers were oriented on the objectives and importance of the study and then asked for consent before being enquired about the HIV status disclosure to their children until the required sample was obtained. During sorting and coding of subjects before analysis, 102 HIV disclosed and 207 nondisclosed participants were identified as shown in Figure 1.

### 2.6. Data Collection and Instruments

Structured modified WHO standard questionnaire translated in Swahili was used. Questionnaires consisted of a series of closed ended questions aimed at capturing necessary information to meet the study objectives. Research Assistants have undergone training on how to administer the questionnaire before data collection. Questions were elaborated and proper interview and writing of caregivers' response were demonstrated. They were blinded about the study to avoid information bias. Using the patients' register in CTC clinics, HIV-infected children between 6 and 17 years on ART for at least six months or more were identified. Assent and consent for the study were obtained from children and their caregivers, respectively. Caregivers who consented for the study were requested to respond to the questions by choosing the correct answer per each question.

### 2.7. Variables

The independent variables included socioeconomic status, parental relationship (biological parents or other), and demographic information of the participants and their guardians.

The dependent variables included HIV status disclosure, treatment adherence, and quality of life.

HIV status disclosure was measured by asking the parents/guardians of the participants the question* “Does the child know his/her HIV status?”* followed by verification of the information with the healthcare providers.

Treatment adherence was measured by using WHO adherence manual, 2007, with the scores categorized as >=95%= GOOD, 85-94%=FAIR, and <85%=POOR. Percentages were computed by the formula: fraction of drug missed per dispensed pills on the last visit*∗*100.

Quality of life was measured by using the 2012 World Health Organization Quality of Life standard tool (WHOQOL-BREF 2012 tool), whereby scores >=80 was considered high quality of life and <80 was considered to be low quality of life. Domains which were used in assessing the quality of life were (i) social relationship which included personal relationships, social support, and sexual activity, (ii) psychological health which included items such as bodily image and appearance, negative feelings, positive feelings, self-esteem, thinking, learning, memory, and concentration, (iii) physical health which included energy, fatigue, pain, discomfort, sleep, and rest, (iv) environmental health which included financial resources, freedom, physical safety and security, health and social care (accessibility and quality), home environment, opportunities for acquiring new information and skills, participation in and opportunities for recreation/leisure, physical environment and transport, and (v) spirituality/religion/personal beliefs which included religion/spirituality/personal beliefs.

### 2.8. Data Analysis

SPSS version 20 was used to process and analyze data. Data were entered into computer software where they were cleaned and analyzed. Descriptive statistics of social demographic characteristics was conducted. Then, Chi square analysis was performed to test for factors related to HIV status disclosure and other outcome variables and adherence to treatment and quality of life, respectively. Variables which showed statistically significant relationship were included in bivariate and multiple logistic regression and p value of 0.05 was used for statistical significance.

### 2.9. Ethical Considerations

Ethical clearance and approval to conduct the study were sought from the University of Dodoma Research and Ethics Committee. Permission to conduct the study in Iringa and Mbeya regions was sought from the Hospital Directors and District Medical Officers. Consent to participate in the study was sought from the parent/guardian of the child before asking for assent from the child. Participants were informed clearly on the aim, risks, and benefits of the study. Caregivers were interviewed in the absence of their children to minimize chances of exposing the child on some of the questions they were not prepared to answer. To ensure confidentiality, the information collected was kept anonymous by not including the names of the participants and their guardians as well as the names of the treatment centres.

## 3. Results

### 3.1. Prevalence of Disclosure

After initial random selection of 309 participants who were included in the analysis, only 102 (33%) had their HIV status disclosed to them. The mean age of participants with disclosed status was 12.39 (SD=3.015) whereas among those with undisclosed status it was 11.29 (SD=3.002). Among those with disclosed HIV status, the majority were in the 14–17-year age group (38.2%), male (51%), and in primary or less education level (63.7%) and had one or both of their biological parents (59.8%). Details of these findings are shown in Table 1.

### 3.2. Factors Associated with HIV Status Disclosure

Chi square analysis as indicated in Table 2 showed that the age of the child (p<0.05), child's level of education (p<0.001), and parent's/guardian's level of education (p<0.05) were significantly related to HIV status disclosure.

Table 3 shows results of bivariate and multiple logistic regression for factors associated with HIV status disclosure. Bivariate logistic analysis showed that, compared to 6 to 9 years of age, the chance of HIV/AIDS status disclosure was 18.3 times higher among children between 10 and 13 years (OR=18.384, CI: 2.449, 138.018) and 64.7 times higher in children between 14 and 17 years (OR=64.755, CI: 8.664, 484.997). Children in secondary level of education had as twice or more odds of HIV status disclosure than those in primary or lower schooling level (OR= 2.846, CI: 1.648, 4.915).

After adjusting for confounders in a multiple logistic regression analysis, findings showed that only the child's age was significantly associated with HIV/AIDS status disclosure. Compared to children in the 6- to 9-year age group, those aged between 10 and 13 years and 14 and 17 years had 19 and 66 (AOR=65.755, p<0.001) times higher odds of HIV status disclosure, respectively.

### 3.3. Association between HIV Status Disclosure and Treatment Adherence

Table 4 shows results from Chi square analysis for the relationship between HIV status disclosure and adherence to ARV treatment. Results showed statistically significant relationship between HIV status disclosure and adherence to ART treatment (p<0.05) whereas age of the child (p<.06) and relationship with the caregiver (p<.07) showed marginal statistical significant relationships.

Table 5 shows unadjusted and adjusted odds ratio for the association between HIV status disclosure and adherence to ARV treatment. Bivariate logistic regression analysis showed only HIV/AIDS status disclosure was significantly associated with ART therapy adherence (p<0.05). The odds of ART adherence was 4.5 times higher among children with HIV status disclosure, compared to those who had no disclosure (OR=4.545, CI: 1.029, 20.071). In the multiple logistic regression, findings showed that HIV/AIDS status disclosure (p<0.05) and being aged between 14 and 17 years of age (p<0.05) were significantly associated with ART adherence. The odds of ART adherence were 8 times higher among children who had HIV status disclosure, as compared to those who had no disclosure of HIV status (AOR = 8.173, p<0.05). With regard to age, being between 14 and 17 years reduced the odds of adhering to treatment (AOR = 0.095 CI: 0.011, 0.850).

### 3.4. Association between HIV Status Disclosure and Quality of Life

Across all domains, quality of life was comparatively high among children with HIV status disclosure compared to those without HIV status disclosure (Figure 2).

Table 6 presents results of Chi square analysis for the relationship between HIV status disclosure and quality of life. Results show that HIV status disclosure (p<0.001), child caregiver relationship (p<0.05), and child's age (<0.05) were significantly related to quality of life. The majority (75.5%) of the participants with HIV status disclosure had a comparatively higher quality of life than those with undisclosed HIV status (49.3%). Quality of life was high (66.4%) among participants living with caregivers other than their biological parents compared to only (46.0%) among children living with their biological parents.

After adjusting for confounders, children with HIV status disclosure had more than three times high odds of having a good quality of life (AOR=3.283, CI: 1.791, 6.017) compared with those with undisclosed status. Children living with their biological parents had half the odds of having a good quality of life (OR=0.500, CI: 0.300, 0.834) compared with those living with a guardian other than their biological parents (Table 7).

## 4. Discussion

The current study aimed at determining factors associated with HIV status disclosure and its effect on treatment adherence and quality of life among children aged 6–17 years in Southern Highlands Zone, Tanzania. In this study, we found that HIV status disclosure was relatively low; only one-third of the participants were aware of their HIV status. We also found that HIV status disclosure was significantly associated with adherence to treatment and high quality of life in children living with HIV/AIDS in a low resource setting.

Since 2011, WHO set up a guideline which recommends HIV status disclosure at the age of 6 years and completed at the age of 12 years [3]. Despite the recommendation, HIV status disclosure to children remains a challenge. Several studies done in Africa and other resource limited settings show low levels of disclosure [5, 10, 11]. The level of HIV status disclosure in children ranges between 8.4 and 79% [5] and from 0 to 69% [6]. Levels of disclosure are much lower in developing countries where HIV in children is even more prevalent. A previous study done in northern Tanzania found the prevalence of HIV status disclosure to be 22.3% [12], a bit lower than the levels reported in the current study. Similar levels have been reported elsewhere in Africa [11, 13, 14]. Parents/caregivers feel uneasy with the disclosure conversation exacerbated by their fear of stigma and discrimination [7]. Limited skills by both parents/guardians and healthcare workers on how to handle the disclosure processes and the uncertainties in the aftermath of disclosure and caring for a child growing up aware of being HIV infected may complicate the situation.

In our study, we found that HIV status disclosure was significantly associated with the age of the child where children aged 10 years and above were more likely to know their HIV status. At the age of 10 years and above, children are on the verge of change in almost all aspects of their lives and become more curious of whatever is going on around them. Similar findings have been reported earlier [11–14]. This could be explained by caregivers' belief that younger children are not mature enough to understand the disease [15, 16] and by the age of 10 years and above parents gain the confidence to disclose HIV status. On the other hand, it takes a time for the provider to build strong trust with the guardians and the child and therefore delaying the time for status disclosure. However, if early disclosure is possible before this age, it makes it easier for the provider to speak with the child regarding the prescribed ARVs, opening room for counselling and health education to the child and the guardian.

In this study, HIV status disclosure was found to be significantly associated with high treatment adherence. Previous studies assessing the association between disclosure and adherence came up with conflicting results. Most of the studies showed that HIV status disclosure improved adherence levels [17–20]. Some studies done to assess barriers to treatment adherence found nondisclosure to be one of the factors [21, 22]. However, some studies have shown a negative association between disclosure and adherence [23, 24].

Studies assessing the association between disclosure and quality of life have come with inconsistent results. Several studies done have found that HIV status disclosure was associated with high quality of life [25, 26]. However, a longitudinal analysis by Butler AM et al. found no association between disclosure and any of the domains of quality of life [27]. In our study, disclosure was significantly associated with quality of life. The differences in findings between studies could be explained by the differences in the measures used for assessing quality of life. They can also be explained by the limited number of study participants and limited data quality to allow for inferential analysis.

## 5. Conclusions and Recommendations

Despite existence of WHO guideline on HIV status disclosure to HIV-infected children and adolescents, prevalence of disclosure was found to be low in this study and often done later after 10 years of age. HIV status disclosure was found to be associated with improved treatment adherence and quality of life irrespective of other factors. Despite the available guideline, how disclosure takes place may vary from culture to culture and from place to place, depending on available resources and caregivers' desires and concerns. There is therefore a need for adapting the guideline to address important local cultural values relevant in sharing and handling sensitive information that involves the lives of children.

## Figures and Tables

**Figure 1:** Showing sampling flow chart.

**Figure 2:** Description of quality of life by domains in relation to HIV status disclosure to children 6-17 years living with HIV/AIDS.

**Table 1:** Distribution of study participants by sociodemographic characteristics (N=309).

**Variable**	**Disclosed**	**Nondisclosed**
	**n (%)**	**n (%)**
Age of the child:		
6–9 years	29 (28.5)	53 (25.6)
10–13 years	34 (33.3)	100 (48.3)
14–17 years	39 (38.2)	54 (26.1)
Sex of the child:		
Female	50 (49)	104 (50.2)
Male	52 (51)	103 (49.8)
Child/caregiver relationships:		
Biological parent(s)	61(59.8)	129 (62.3)
Others	41(40.2)	78 (37.7)
Child's level of education:		
Primary or less	65 (63.7)	171(82.6)
Secondary or higher	37 (36.3)	36 (17.4)
Caregiver level of education:		
Primary or less	5 (4.9)	25 (12.1)
Secondary or high	97 (95.1)	182 (87.9)
Caregiver income:		
Employment	70 (68.6)	135 (65.2)
Others	32 (31.4)	72 (34.8)

**Table 2:** Factors related with HIV status disclosure, among children between 6 and 17 years on ART, in Southern Highlands Zone, Tanzania (N=309).

**Variable**	**HIV status disclosure**				**P value**
	**Undisclosed (n=207)**		**Disclosed (n=102)**		
	**N**	%	**N**	%	
Age of the child:					
6–9 years	53	64.6	29	35.4	
10–13 years	100	74.6	34	25.4	<0.05
14–17 years	54	58.1	39	41.9	
Child's sex:					
Males	104	67.5	50	32.5	0.840
Females	103	66.5	52	33.5	
Child/caregiver relationship:					
Biological parents	128	67.7	61	32.3	0.730
Others	79	65.8	41	34.2	
Child's level of education:					
Primary or less	173	72.7	65	27.3	<0.001
Secondary or high	34	47.9	37	52.1	
Caregiver level of education:					
Primary or less	155	70.5	65	29.5	<0.05
Secondary or high	52	58.4	37	41.6	
Caregiver income:					
Employment	55	61.1	35	38.9	0.159
Others	152	69.4	67	30.6	

**Table 3:** Crude and adjusted odds ratio for factors associated with HIV status disclosure, among children between 6 and 17 years on ART therapy, in Southern Highlands Zone, Tanzania (N=309).

**Variables**	**OR**	**95% CI**	**P value**	**AOR**	**95% CI**	**P value**
Age of child:						
6–9 years	Ref					
						
10–13 years	18.384	2.449, 138.018	<0.01	19.178	2.535, 145.102	<0.05
14–17 years	64.755	8.664, 483.997	<0.001	65.723	8.463, 510.421	<0.001
Child's level of education:						
Primary or less	Ref					
Secondary or high	2.846	1.648, 4.915	<0.001	0.966	0.519, 2.098	0.904
Caregiver level of education:						
Primary or less	Ref					
Secondary or high	1.664	0.997, 2.776	0.051	1.125	0.601, 2.107	0.713

**Table 4:** Relationship between HIV status disclosure and ART adherence, among children between 6 and 17 years on antiretroviral therapy, in Southern Highlands Zone, Tanzania (N=309).

**Variable**	**ART adherence**		**P value**
	**Adherent** **n (%)**	**Nonadherent** **n (%)**	
Age of child:			
6–9 years	3 (3.7)	79 (96.3)	
10–13 years	7 (5.2)	127 (94.8)	0.063
14–17 years	11 (11.8)	82 (88.2)	
HIV status disclosure:			
No	19 (9.2)	188 (90.8)	<0.05
Yes	2 (2.0)	100 (98.0)	
Child's sex:			
Male	10 (6.5)	144 (93.5)	0.833
Female	11(7.1)	144 (92.9)	
Child/caregiver relationship:			
Biological parents	9 (4.8)	180 (95.2)	0.075
Others	12 (10.0)	108 (90.0)	
Caregiver income			
Employment	7 (7.8)	83 (92.2)	0.660
Others	17 (6.4)	205 (93.6)	
Ever hospitalized:			
Yes	13 (6.4)	190 (93.6)	0.705
No	8 (7.5)	98 (92.5)	
Child's level of education:			
Primary or less	15 (6.3)	223 (93.7)	0.528
Secondary or high	6 (8.5)	65 (91.5)	
Caregiver level of education:			
Primary or less	17 (7.7)	203 (92.3)	0.307
Secondary or high	4 (4.5)	85 (95.5)	

**Table 5:** Crude and adjusted analysis for the association between HIV status disclosure and ART adherence, among children between 6 and 17 years on antiretroviral therapy in Southern Highlands Zone, Tanzania (N=309).

**Variables**	**OR (95% CI)**	**P value**	**AOR (95% CI)**	**P value**
HIV status disclosure:				
No	Ref			
Yes	4.545(1.029, 20.071)	<0.05	8.173(1.765, 37.842)	<0.05
Age of child:				
6 – 9 years	Ref			
10–13 years	0.349(2.042, 2.907)	0.330	0.288(0.034, 2.423)	0.252
14-17 years	0.189(0.024, 1.502)	0.115	0.095(0.011, 0.850)	<0.05
Caregivers education:				
Primary or less	Ref			
Secondary or high	1.578(0.509, 4.893)	0.430	1.825(0.543, 6.138)	0.331

**Table 6:** Relationship between HIV status disclosure and quality of life, among children between 6 and 17 years on antiretroviral therapy, in Southern Highlands Zone, Tanzania (N=309) Chi square.

**Variable**	**Quality of Life**		**P value**
	**Low** **n (%)**	**High** **n (%)**	
HIV status disclosure:			
No	102 (49.3)	105 (50.7)	<0.001
Yes	25 (24.5)	77 (75.5)	
Child/caregiver relationship:			
Biological parents	87 (46.0)	102 (54.0)	<0.05
Others	40 (33.3)	80 (66.7)	
Sex of the child:			
Males	69 (44.8)	85 (55.2)	0.187
Females	58 (37.4)	97 (62.60	
Age of the child:			
6 to 9 years	30 (55.6)	24 (44.4)	<0.05
10 to 13 years	54 (40.0)	81 (60.0)	
14 to 17 years	43 (35.8)	77 (64.2)	

ART adherence:	10 (47.6)	11(52.4)	0.529
No	117 (40.6)	171(59.4)	
Yes			
Caregiver income			
Employment	40 (44.4)	50 (55.6)	
Others	87 (39.7)	132 (60.3)	0.444
Child's level of education:			
Primary or less	99 (41.6)	139 (58.4)	0.745
Secondary or high	28 (39.4)	43 (60.6)	
Caregiver level of education:			
Primary or less	87 (39.5)	133 (60.5)	0.382
Secondary or high	40 (44.9)	49 (55.1)	

**Table 7:** Crude and adjusted ratio for the association between HIV status disclosure and quality of life, among children between 6 and 17 years on ART, in Southern Highlands Zone, Tanzania (N = 309).

**Variables**	**OR (95% CI)**	**P value**	**AOR (95% CI)**	**P value**
HIV status disclosure:				
No	Ref			
Yes	3.203 (1.889, 5.432)	<0.001	3.283(1.791, 6.017)	<0.001
Age of the child:				
6 to 9 years	Ref			
10 to 13 years	2.165 (1.353, 3.464)	0.111	1.403 (0.709, 2.776)	0.331
14 to 17 years	2.060 (1.068, 3.971)	<0.05	1.513 (0.656, 3.485)	0.331
Sex of the child				
Males	Ref			
Females	1.451 (0.920, 2.289)	0.110	1.602 (0.978, 2.625)	0.061
Child/caregiver relationships:				
Biological parent(s)	Ref			
Others	1.796 (1.114, 2.888)	0.016	0.500 (0.300, 0.834)	<0.05
ART adherence:				
No	Ref			
Yes	1.569 (0.619, 3.978)	0.343	1.567 (0.578, 4.249)	0.378

## Data Availability

The datasets analyzed during the current study are available from the corresponding author on reasonable request.

## Abbreviations

AIDS: Acquired Immune Deficiency Syndrome
AOR: Adjusted odds ratio
ART: Antiretroviral treatment
ARV: Antiretroviral
CTC: Care and treatment centre
GHSS: Global health sector strategy
HAART: Highly active antiretroviral therapy
HIV: Human immunodeficiency virus
HTC: HIV testing and counselling
HRQOL: Health-related quality of life
MTCT: Mother to child transmission
NBS: National Bureau of Standards
NACP: National AIDS Control Programme
OIs: Opportunistic infections
OR: Odds ratio
PCP: Pneumocystis carinii pneumonia
PMTCT: Prevention of mother to child transmission of HIV
QOL: Quality of life
SD: Standard deviation
SPSS: Statistical package for the social sciences
SRS: Simple random sampling
TB: Tuberculosis
THMIS: Tanzania Health Management Information System
UNAIDS: United Nations Programme on HIV/AIDS
USAID: United States Agency for International Development
UNICEF: United Nations Children's Fund
VCT: Voluntary, counselling, and testing
WHO: World Health Organization.
